The article "Evaluation of the reduction of radiation dose received by pediatric patients in new-generation biplane angiocardiography: Randomized controlled study" was published in 2024. Journal: Heliyon.

# Evaluation of the reduction of radiation dose received by pediatric patients in new-generation biplane angiocardiography: Randomized controlled study

**DOI:** 10.1016/j.heliyon.2024.e28138

**Published:** 2024-03-22

**Authors:** Osman Başpınar, Mehmet Kervancıoğlu, Metin Kılınç, Derya Aydın Şahin, Münevver Tuğba Temel

**Affiliations:** Gaziantep University, Faculty of Medicine, Department of Pediatric Cardiology, Turkey

**Keywords:** Patent ductus arteriosus, Transcatheter occlusion, Radiation, Dose area product, Air kerma, Childhood

## Abstract

**Objective:**

We aimed to evaluate the safety and efficacy of radiation dose reduction with a new-generation biplane angiocardiography system in patients undergoing transcatheter isolated patent ductus arteriosus (PDA) closure.

**Materials and methods:**

Fifty pediatric patients who underwent transcatheter PDA closure were randomly divided into two groups as normal radiation dose and low dose. Patients who required additional procedures other than PDA closure were excluded. PDA closure was performed according to the angiographic measurement of the defect. After the procedure, age, weight, sex, PDA measurements, and radiation measurements such as dose-area product (DAP, Gy.cm^2^) and air kerma (AK, mGy) were compared between the groups.

**Results:**

There was no statistically significant difference between the groups in age, sex, weight, PDA diameter, PDA type, device used, and device diameter (p > 0.05). While there was no statistically significant difference between the groups in terms of cine recording, number of recorded images, and fluoroscopy time (p > 0.05), there was a statistically significant difference between the total DAP, cine and fluoroscopy DAP, total AK, frontal and lateral tube AK, and DAP/kg (mGy.m^2^/kg) measurements (p < 0.05).

**Conclusion:**

Transcatheter PDA closure with a low radiation dose is as effective as that with a normal radiation dose. The radiation dose received by the patient during the procedure was significantly reduced. With the vision provided by this study, it seems possible to work with a low radiation dose in other groups of patients.

## 1 Introduction

The occurrence of cancer due to radiation doses and stochastic effects is well known. This is even more important for children with a long-life expectancy. It highlights the importance of the as low as reasonably achievable (ALARA) principle, which should be considered in diagnostic or interventional cardiac catheterization for congenital heart disease [[1], [2], [3], [4]]. Repeated cardiac catheterizations, chest radiographs, and computed tomography scans are required in children with congenital heart disease, especially in complex diseases. Shortening the duration of cine cardiography during each catheterization procedure alone is not sufficient to reduce the dose. In addition, it is recommended to acquire the fluoroscopic image instead of the cine image, to use collimation, not to make recordings of unnecessary areas for too long, and to optimize the distance of the detector from the patient [[1], [2], [3], [4]]. In our study, we evaluated the efficiency of the procedure and the success of dose reduction with a randomized method in transcatheter closure of the patent ductus arteriosus (PDA) by dose reduction using the ClarityIQ program of the Philips Azurion 7 B20/12® (Philips Medical Systems, Eindhoven, The Netherlands) angiocardiography system.

The article "Evaluation of the reduction of radiation dose received by pediatric patients in new-generation biplane angiocardiography: Randomized controlled study" was published in 2024. Journal: Heliyon.

The deterministic and stochastic effects of radiation were determined by measurements of dose-area product (DAP, Gy.cm^2^) and air Kerma (AK, mGy). Low and normal dose were compared in terms of effectiveness and radiation doses. The deterministic effect is related to the cell damage caused by radiation. It occurs when the radiation dose exceeds a certain threshold. When the threshold is exceeded, the severity of tissue reactions increases with increasing radiation dose. The threshold dose is usually 2 Gy for transient skin redness and 3 Gy for transient hair loss. Air Kerma is used to determine the deterministic effects of ionizing radiation. Stochastic effects refer to mutations caused by DNA damage that can occur at low levels of radiation. In the long term, cancer may develop. It is maintained that the stochastic risk, or probability of developing cancer, is directly proportional to the total radiation dose received and there is no threshold as in deterministic risk. Dose-area product is used to estimate the risk of stochastic effects [[5], [6], [7], [8]].

As a function of the new-generation angiocardiography system (Philips Azurion 7®), a dose model is created after the procedure [9]. In this modeling, the thoracic region is represented as a sphere with a diameter of 30 cm arranged around the isocenter. The surface of this sphere is divided into 10 areas, five on the cranial and five on caudal sides, corresponding to the different projections of the X-ray beam [9]. In the dose model and report, in addition to the fluoroscopy time, the number of series, the number of images, the total DAP, the cine DAP, the fluoroscopy-induced DAP, the total cumulative AK of the whole body, the real cumulative peak AK of the hottest spot in the irradiated body region, and the frontal and lateral tube AK are indicated numerically and graphically [9]. (Fig. 1, Fig. 2.). In addition, a warning is given when the peak AK in the irradiated body region is above the threshold (2 Gy).

The article "Evaluation of the reduction of radiation dose received by pediatric patients in new-generation biplane angiocardiography: Randomized controlled study" was published in 2024. Journal: Heliyon.

**Fig. 1:** First page of Philips Azurion 7 biplane angiocardiography device dose model one of a patient from low dose group. DAP total dose, cine and fluoroscopy DAP, AK total dose, and AK dose for frontal and lateral tube are given in Gy.cm^2^ and mGy. In addition, the number of series, number of images, and what part of the thorax receives the maximum AK dose through which tube are shown in the figure. (DAP, dose-area product; AK, air kerma).

**Fig. 2:** Second page of the Philips Azurion 7 biplane angiocardiography device dose model one of a patient from low dose group. DAP, total AK, and frontal and lateral AK doses are given in Gy.cm^2^ and mGy per dose. The number of series, number of images, and number of images per second are also shown. (DAP, dose-area product; AK, air kerma).

## 2 Material

### 2.1 Research method

A total of 50 children undergoing isolated transcatheter closure of the PDA were randomly divided into two separate groups of 25 to ensure homogeneity of the patient group. Both groups were treated using the same biplane angiocardiography machine, one group with normal radiation dose and the other group with low radiation dose using the new-generation ClarityIQ program. Patients who underwent aortic/pulmonary balloon valvuloplasty, or aortopulmonary collateral artery occlusion in the same session and patients with complicated additional procedures that required a longer procedure time were excluded from the study. For standardization, the frame per second (fps) number was kept at the recommended fixed 25 fps.

### 2.2 Measurements and parameters monitored

Patient demographics included sex, age, height, and weight. During PDA closure, defect type, length, ampulla diameter, pulmonary tip diameter, pulmonary artery pressure, shunt ratio, device type, and device size were detected. Angiographic images of each patient and contrast injection were obtained in the standard right anterior oblique (RAO) and lateral positions. After the occlusion procedure, the efficacy of the procedure was evaluated with a control contrast injection in the RAO and lateral positions. Fluoroscopy time, total DAP, cine DAP, fluoroscopy DAP, total AK, separate AK of the frontal and lateral tubes, and peak AK were recorded in the automatic radiation measurement report of the angiography machine. DAP (Gy.cm^2^) was converted to mGy.m^2^ and indexed as DAP/kg.

### 2.3 Data analysis

Patients were randomly divided into two groups: a normal standard-dose and a low-dose group. Demographic data are expressed as percentage, mean, median, standard deviation, minimum-maximum value, and interquartile range (IQR). Analyses were performed using the SPSS 22.0 program. Demographic characteristics of the participants are presented as frequency and percentage. Parametric measurements were compared using the *t*-test for independent groups and nonparametric measures were compared using the one-way analysis of variance. Percentages were analyzed using the chi-square test. A value of P < 0.05 was considered statistically significant.

The article "Evaluation of the reduction of radiation dose received by pediatric patients in new-generation biplane angiocardiography: Randomized controlled study" was published in 2024. Journal: Heliyon.

### 2.4 Ethics Committee approval

Ethics committee approval was obtained. Written informed consent forms were obtained from the patients' families and patients who were old enough to provide their consent for participation in the study.

### 2.5 Study schedule

This study was conducted between December 2021 and October 2022 with patients who applied to our pediatric cardiology outpatient clinic and underwent PDA closure.

The system used was Philips Azurion 7 B20/12® model. The radiation protocol was selected as normal and low with the ClarityIQ® system of the device.^9^ Special filters in the ionizing radiation tube, kV and mA values were changed and normal and low-dose radiation adjustments could be made according to the body surfaces and weights of the patients. With the technological advantages offered by ClarityIQ, 500 parameters can be fine-tuned to reduce noise, sharpen edges, increase filtering, reduce focusing, change the grid, and enable the tube and generator to deliver a shorter pulse current. In addition, the Zero Dose Positioning® system in Philips angiography devices allows the patient's image focus to be changed without the use of fluoroscopy; the Last Image Hold® feature allows the last fluoroscopy images to be recorded and DoseAware® is a protective measure that allows the patient and staff to receive less dose. Radiation measurement parameters vary depending on the technique. Measurements in this study were Gray (Gy), along with dose area product of Gy.cm^2^. AK is the amount of kinetic energy released into the air due to ionizing radiation, expressed in mGy, where 1 Gy = 1 J/kg. Peak AK is the highest AK value to which any point of a surface exposed to radiation is exposed. Skin dose is the absorbed dose delivered by ionizing radiation to the patient's skin at the point of irradiation. Unlike the reference AK, this value determines the actual absorption. DAP is the product area cross-section of the X-ray beam and the AK value averaged over this cross-section, expressed in Gy.cm^2^. Unlike skin dose and AK, DAP is independent of the distance from the focal point. The unit of measurement is converted to mGy.m^2^ by multiplying by 100 for comparison with other studies. It was also indexed by dividing by weight and DAP/kg, and mGy.m^2^/kg was obtained.

The article "Evaluation of the reduction of radiation dose received by pediatric patients in new-generation biplane angiocardiography: Randomized controlled study" was published in 2024. Journal: Heliyon.

## 3 Results

### 3.1 Demographic characteristics of the participants

Twenty-eight (56%) of the 50 patients were female with a mean weight of 8.6 ± 7.1 (3.3–35) kg. The arterial and venous sheaths were inserted in 32 patients (64%), and the most common form of PDA was type A conical type. The mean pulmonary artery pressure was 25 ± 12.9 (12–65) mmHg. The PDA at the pulmonary artery end was 2.2 ± 1.0 (1–4.9) mm and the shunt ratio was 1.6 ± 1.1 (1–5.8). When patients were randomly divided into two groups (normal and low dose), there was no statistically significant difference between demographic data, and the groups were homogeneous (p > 0.05, Table 1.).

**Table 1:** Comparison of patient groups demographic characteristics divided into low and normal radiation dose.

Data	Overall result	Low dose	Normal dose	p
Age (years)	1 ± 2.9 (0.2–10.6)	2.7 ± 2.9 (0.2–9.6)	2.3 ± 2.9 (0.3–10.6)	0.702
Sex	28 F (56%)	13 M (52%)	16 F (64%)	0.264
Weight (kg)	8.6 ± 7.1 (3.3–35)	11.3 ± 6.7 (3.3–35)	10.7 ± 7.7 (4.6–33)	0.785
Body surface (m^2^)	0.4 ± 0.2 (0.2–1.1)	0.5 ± 0.2 (0.2–1.1)	0.4 ± 0.2 (0.2–1.1)	0.705
Access	32 arteries and veins (64%), 18 isolated arteries (36%)	15 arteries and veins (60%), 10 arteries (40%)	17 arteries and veins (68%), 8 arteries (32%)	0.556
Mean pulmonary artery pressure (mmHg)	25 ± 12.9 (12–65)	27.1 ± 10.3 (16–65)	28.8 ± 15.6 (14–63)	0.670
PDA type	29A (34%), 14E (28%), 4C, 3D	16A, 7E, 1C, 1D	13A, 7E, 3C, 2D	0.590
PDA pulmonary diameter (mm)	2.2 ± 1 (1–4.9)	2.4 ± 0.8 (1.2–4.3)	2.3 ± 1.1 (1.5–4.9)	0.678
PDA ampulla diameter (mm)	7.4 ± 3.2 (1.1–19.5)	8.6 ± 3.2 (3.8–19.5)	7.5 ± 3.2 (4–15)	0.289
PDA length (mm)	8.9 ± 3.6 (2.9–18.2)	10.3 ± 4.3 (2.9–18.2)	8.7 ± 2.7 (5.7–13.5)	0.112
Shunt ratio	1.6 ± 1.1 (1–5.8)	1.9 ± 1.2 (1–5.8)	1.9 ± 1.0 (1.3–4.9)	0.858
Device type	22 APO (44%), 17 ADO (34%), 8 ADO2, 3 MVSD	9 ADO (36%), 8 APO (32%), 7 ADO2, 1 MVSD	14 APO (56%), 8 ADO (32%), 2 MVSD, 1 ADO2	0.204
Device diameter	Most common ADO 8/6 in 13	Most common ADO 8/6 in 7	Most common ADO 8/6 in 6	0.650
Delivery route	28 retrograde (56%)	14 retrograde	14 retrograde	1.00

PDA, patent ductus arteriosus, according to PDA type A, B, C, D, and E classification; APO, Amplatzer Piccolo Occluder; ADO, Amplatzer Ductal Occluder; ADO2, Amplatzer Ductal Occluder Type 2; MVSD, Amplatzer Muscular Ventricular Septal Defect Occluder.

The method of vascular access, PDA type, PDA size, pulmonary artery pressure, shunt ratio, device types and diameters used, and device delivery ways were assessed in the cardiac catheterization of patients who received low- and normal-dose radiation. No difference was found between the groups regarding the measured parameters (p > 0.05, Table 1.). Down syndrome was detected in six patients and pulmonary hypertension in 11 patients. Transcatheter PDA closure was successfully performed in all patients in each group without residual shunts and iatrogenic the left pulmonary artery and aortic obstructions. There were no major complications between groups, and the minor complications (hematoma at the enterance point, transient hypoxemia during sedation, transient arrhythmias) were not related to assigned radiation dose.

The article "Evaluation of the reduction of radiation dose received by pediatric patients in new-generation biplane angiocardiography: Randomized controlled study" was published in 2024. Journal: Heliyon.

After cardiac catheterization, patients' dose reports were automatically appended to the end of the cine images, and dose models were created. An example of the dose report of one of our patients is shown in Fig. 1, Fig. 2.

While there was no statistically significant difference between the number of series and images and fluoroscopy duration among the low- and normal-radiation dose groups (p > 0.05), a significant difference was observed between total DAP, cine DAP, fluoroscopy DAP, total AK, frontal AK, and lateral AK measurements (p < 0.05) (Table 2, Fig. 3, Fig. 4.).

**Table 2:** Comparison of automatic dose measurement parameters of patients receiving low- and normal-dose radiation.

Data	Total	Low dose	Normal dose	p
Total DAP (Gy.cm^2^)	0.8 ± 0.6 (0.1–3.1)	0.5 ± 0.3 (0.1–1.6)	1.1 ± 0.8 (0.3–3.1)	0.002*
Total DAP (mGy.m^2^)	85.7 ± 67.5 (14.3–316.6)	57 ± 34.3 (14.3–161.5)	114.4 ± 80.1 (32.9–316.6)	0.002*
Cine DAP (Gy.cm^2^)	0.1 ± 0.1 (0.03–0.7)	0.1 ± 0.08 (0.03–0.3)	0.2 ± 0.1 (0.07–0.7)	0.001*
Fluoroscopy DAP (Gy.cm^2^)	0.6 ± 0.5 (0.1–2.9)	0.4 ± 0.2 (0.1–1.3)	0.8 ± 0.7 (0.2–2.9)	0.006*
DAP/kg (mGy.m^2^/kg)	8.6 ± 6.8 (1.6–23.4)	5.6 ± 3.6 (1.6–17.9)	11.6 ± 5.7 (4.6–23.4)	0.000*
Total AK (mGy)	10 ± 8.3 (2.2–51.7)	6.3 ± 3.3 (2.2–17.8)	13.7 ± 10.1 (5–26.8)	0.001*
Frontal AK (mGy)	2.5 ± 1.7 (0.4–9.9)	1.8 ± 1.1 (0.6–4.2)	3.2 ± 2 (1.4–9.9)	0.003*
Lateral AK (mGy)	7.4 ± 7.9 (1.4–51.2)	4.5 ± 2.8 (1.4–13.9)	10.4 ± 10 (3.4–16.9)	0.006*
Total number of series	3.2 ± 1.3 (2–7)	3.2 ± 1.5 (2–7)	3.3 ± 1 (2–5)	0.749
Number of images	376 ± 176.1 (162–968)	346 ± 149.9 (195–699)	407.5 ± 197.1 (189–968)	0.221
Fluoroscopy time (min)	4.3 ± 2.4 (1.6–15)	4 ± 2 (1.6–10.9)	4.6 ± 2.8 (2–9.9)	0.442

DAP; dose-area product, dose area product, AK; air Kerma, * statistically significant.

**Fig. 3:** Boxplot with linear scales of total, cine, and fluoroscopic DAP measurements in patients who received low or normal doses of ionizing radiation during PDA closure (p < 0.05). (DAP, dose-area product; PDA, patent ductus arteriosus).

**Fig. 4:** Boxplot with power scales of total, frontal, and lateral AK measurements in patients who received a low or normal dose of ionizing radiation during PDA closure (p < 0.05). (AK, air kerma; PDA, patent ductus arteriosus).

The article "Evaluation of the reduction of radiation dose received by pediatric patients in new-generation biplane angiocardiography: Randomized controlled study" was published in 2024. Journal: Heliyon.

Measurements of DAP/kg (mGy.m^2^/kg) and calculations to standardize DAP values to patient weight were performed in both groups, and there was a statistically significant difference between measurements (mean 5.6 ± 3.6 [1.6–17.9] vs. mean 11.6 ± 5.7 [4.6–23.4], p < 0.0001) (Table 2 and Fig. 5). The median low DAP dose/kg was 4.68 (IQR 3.2 and 6.89) and the median AK was 5.53 (IQR 4.2 and 7.7). We found that the highest radiation dose was from the lateral exposure in 48 patients and from the frontal tube in only two patients.

**Fig. 5:** Comparison of patients receiving low and normal dose of ionizing radiation after standardization of DAP showing stochastic effect of radiation with weight (DAP/kg, mGy.m^2^/kg; p < 0.001). (DAP, dose-area product; 1, low dose; 2, normal dose).

## 4 Discussion

Especially in children with complex congenital heart disease, ionizing radiation exposure increases with repeated cardiac catheterization. To protect the cardiology staff and the pediatric patient, the ALARA principle is often implemented. Other practices include using flat-panel detectors, avoiding unnecessary imaging, shortening fluoroscopy time, using nonradioactive methods such as echocardiography whenever possible, using fluoroscopy recordings instead of cine recordings, using collimation, and keeping the detector close to the patient [[1], [2], [3], [4], [5], [6], [7], [8]]. In pediatric patients, the number of fps is higher than in adults because of the higher heart rate, but it may be possible to reduce fps significantly, especially for procedures such as transcatheter closure of secundum atrial septal defects [10,11].

The harmful effect of radiation depends on the dose received by the patient; therefore, dose reduction is critical. Although the stochastic effect is independent of the threshold dose, its frequency is expected to increase with increasing dose [[12], [13], [14]]. In our study, the number of fps was kept constant according to the general recommendation for children to determine the effect of dose reduction, while the dose of ionizing radiation was adjusted as normal and low dose. It was found that the use of low-dose radiation made a statistically significant difference in the DAP and AK units in which the risk of deterministic and stochastic effects was measured, while not resulting in a decrease in success. The randomized selection of groups, the selection of a procedure such as transcatheter PDA closure that requires homogeneity, the standardized use by a single physician, and the prospective study design are the positive aspects of the study.

The Philips AlluraClarity® radiation dose reduction system was found to be efficient and effective by Bracken et al. [15] in 268 patients with coronary artery disease and by Sullivan et al. [8] in 430 pediatric patients, with the previous version of ClarityIQ. The newly developed system was evaluated in our study and resulted in significant DAP and AK reduction even when fps was maintained at the standard level.

The article "Evaluation of the reduction of radiation dose received by pediatric patients in new-generation biplane angiocardiography: Randomized controlled study" was published in 2024. Journal: Heliyon.

AK and DAP measurements can be used to determine the deterministic and stochastic adverse effects of radiation. It is even more important that this can be achieved without compromising the success and without reducing the number of fps, which is an important indicator of image quality. Studies find that partially reducing the number of fps, further reduces the amount of radioactivity. Because image sharpness is even less important in transcatheter closure of a secundum atrial septal defect, the number of fps can even be reduced to single digits [4,[10], [11], [12]]. However, as was the case with the present study, the fps number may need to be kept higher because measurement of the diameters and length of the PDA is critical for proper device selection.

When DAP/kg was standardized, the results of our study were found to be significantly lower compared with other studies. To allow objective comparison with these studies, transcatheter PDA closure and median DAP (mGy.m^2^/kg) and median AK (mGy) and interquartile measurements were used as units of measurement. Ghelani et al. [16], first published national radiation doses in 2014. In 2017, the results were updated with more than 2000 cases from seven centers.^2^ Patel et al. [14] obtained the lowest DAP/kg and AK measurements for six different procedures, particularly atrial septal defect and PDA closure. In addition to these large studies, smaller studies by Borik et al. [12] achieved dose reductions of approximately 50% in atrial septal defect and PDA closure at 7.5 fps. Kyobashi et al. [17] demonstrated low DAP in a study that was not indexed by patient body weight. Compared with these studies, our study was able to achieve the lowest DAP/kg and AK values by keeping not lowering fps numbers (Table 3). It was found that the fine-tuning of the ClarityIQ program was quite efficient. After this phase, a same or similar study should be performed by decreasing the number of fps to reach the lowest effective radiation dose.

**Table 3:** Comparison of our study and other studies on ionizing radiation reduction during transcatheter PDA closure (median values).

	Our study	Borik [12]	Patel [14]	Kyobashi [17]	Hirshfeld [18]	Glatz [19]
DAP/kg	4.7*	18	24	42	37	352†
AK	5.5*	–	23	–	73	–

DAP, dose-area product; AK, air kerma, * lowest median ionizing radiation values, † did not index DAP to weight.

The article "Evaluation of the reduction of radiation dose received by pediatric patients in new-generation biplane angiocardiography: Randomized controlled study" was published in 2024. Journal: Heliyon.

In 48 patients, it was observed that the highest value of the AK dose was caused by lateral exposure and only in two patients by RAO exposure originating from the frontal tube. This finding supports that highest radiation scattering measurements with biplane angiographic tubes are most often associated with excessive angulation of the lateral tube [20].

A limitation of our study may be that we did not reduce the fps numbers. Although we could certainly achieve lower radiation values by reducing the frame rate, it would not have been possible to determine the effectiveness of the ClarityIQ system.

## Ethics Committee approval

Ethical committee approval was received from the Ethics Committee of Gaziantep University (Decision No: 25/2019).

## Funding

This research supported by 10.13039/501100008836Gaziantep University research funding.

## Data availability statement

Data available at Gaziantep University electronic data bank.

## Informed consent

Written informed consent was obtained from all participants who participated in this study.

## CRediT authorship contribution statement

**Osman Başpınar:** Writing – review & editing, Writing – original draft, Visualization, Supervision, Project administration, Methodology, Investigation, Funding acquisition, Data curation. **Mehmet Kervancıoğlu:** Supervision. **Metin Kılınç:** Visualization. **Derya Aydın Şahin:** Data curation. **Münevver Tuğba Temel:** Validation.

## Declaration of competing interest

The authors declare that they have no known competing financial interests or personal relationships that could have appeared to influence the work reported in this paper.

## References

[1] Agarwal S., Parashar A., Bajaj N.S. (2014). Relationship of beam angulation and radiation exposure in the cardiac catheterization laboratory. JACC Cardiovasc. Interv..

[2] Cevallos P.C., Rose M.J., Armsby L.B. (2016). Implementation of methodology for quality improvement in pediatric cardiac catheterization: a multicenter initiative by the congenital cardiac catheterization project outcomes quality improvement (C3PO-QI). Pediatr. Cardiol..

[3] Ahmed T.A.N., Taha S. (2017). Radiation exposure: the forgotten enemy: toward implementation of national safety program. Egypt Heart J..

[4] Sitefane F., Malekzadeh-Milani S., Villemain O., Ladouceur M., Boudjemline Y. (2018). Reduction of radiation exposure in transcatheter atrial septal defect closure: how low must we go?. Arch. Cardiovasc. Dis..

[5] Heidbuchel H., Wittkampf F.H.M., Vano E. (2014). Practical ways to reduce radiation dose for patients and staff during device implantations and electrophysiological procedures. Europace.

The article "Evaluation of the reduction of radiation dose received by pediatric patients in new-generation biplane angiocardiography: Randomized controlled study" was published in 2024. Journal: Heliyon.

[6] Manu S., Suntharos P., Boyle G.J., Wang L., Prieto L.R. (2018). Radiation reduction in the pediatric catheterization laboratory using a novel imaging system. J. Invasive Cardiol..

[7] Lamers L.J., Morray B.H., Nugent A., Speidel M., Suntharos P., Prieto L. (2019). Multicenter assessment of radiation exposure during pediatric cardiac catheterizations using a novel imaging system. J. Intervent. Cardiol..

[8] Sullivan P.M., Harrison D., Badran S., Takao C.M., Ing F.F. (2017). Reduction in radiation dose in pediatric cardiac catheterization lab using the Philips AlluraClarity X-ray system. Pediatr. Cardiol..

[9] aaaaa https://www.philips.ro/healthcare/resources/landing/azurion/articles/clarityiq. Accessed 26.December.22.

[10] Gokalp S., Tanidir I.C., Ozturk E., Ergul Y., Guzeltas A. (2021). Radiation dose reduction in congenital heart disease patients during cardiac catheterization by a novel protocol. Turk. Arch. Pediatr..

[11] Tanidir I.C., Gokalp S., Ozturk E., Cilsal E., Topkarci M.E., Guzeltas A. (2020). Is it possible to reduce radiation exposure during transcatheter atrial septal defect closure in children?. Turk Kardiyol. Dernegi Arsivi.

[12] Borik S., Devadas S., Mroczek D., Lee K.J., Chaturvedi R., Benson L.N. (2015). Achievable radiation reduction during pediatric cardiac catheterization: how low can we go?. Cathet. Cardiovasc. Interv..

[13] Quinn B.P., Armstrong A.K., Bauser-Heaton H.D. (2019). Radiation risk categories in cardiac catheterization for congenital heart disease: a tool to aid in the evaluation of radiation outcomes. Pediatr. Cardiol..

[14] Patel C., Grossman M., Shabanova V., Asnes J. (2019). Reducing radiation exposure in cardiac catheterizations for congenital heart disease. Pediatr. Cardiol..

[16] Ghelani S.J., Glatz A.C., David S. (2014). Radiation dose benchmarks during cardiac catheterization for congenital heart disease in the United States. JACC Cardiovasc. lnterv..

[17] Kobayashi D., Meadows J., Forbes T.J. (2014). Standardizing radiation dose reporting in the pediatric cardiac catheterization laboratory, a multicenter study by the CCISC (congenital cardiovascular interventional study consortium). Cathet. Cardiovasc. Interv..

[18] Hirshfeld J.W., Balter S., Brinker J.A. (2004). ACCF/AHA/HRS/SCAI clinical competence statement on physician knowledge to optimize patient safety and image quality in fluoroscopically guided invasive cardiovascular procedures: a report of the American College of Cardiology Foundation/American Heart Association/American College of Physicians Task Force on clinical competence and training. J. Am. Coll. Cardiol..

[19] Glatz A.C., Patel A., Zhu X. (2014). Patient radiation exposure in a modern, large-volume, pediatric cardiac catheterization laboratory. Pediatr. Cardiol..

The article "Evaluation of the reduction of radiation dose received by pediatric patients in new-generation biplane angiocardiography: Randomized controlled study" was published in 2024. Journal: Heliyon.

[20] Bashore T.M., Balter S., Barac A. (2012). American college of cardiology foundation/society for cardiovascular angiography and interventions expert consensus document on cardiac catheterization laboratory standards update: a report of the American college of cardiology foundation task force on expert consensus documents developed in collaboration with the society of thoracic surgeons and society of vascular medicine. J. Am. Coll. Cardiol..

[20] Bracken J.A., Mauti M., Kim M.S., Messenger J.C., Carroll J.D. (2015). A radiation dose reduction technology to improve patient safety during cardiac catheterization interventions. J. Intervent. Cardiol..

